# Applying analytic hierarchy process and failure likelihood index method (AHP-FLIM) to assess human reliability in critical and sensitive jobs of a petrochemical industry

**DOI:** 10.1016/j.heliyon.2022.e09509

**Published:** 2022-05-21

**Authors:** Asma Zare, Naser Hoboubi, Salman Farahbakhsh, Mehdi Jahangiri

**Affiliations:** a Department of Occupational Health Engineering, Sirjan School of Medical Sciences, Sirjan, Iran; b Student Research Committee, Department of Occupational Health Engineering, Shiraz University of Medical Sciences, Shiraz, Iran; c Research Center for Health Sciences, Department of Occupational Health Engineering, School of Health, Shiraz University of Medical Sciences, Shiraz, Iran

**Keywords:** Human reliability assessment, Human error, Petrochemical industry, AHP-FLIM

## Abstract

**Background:**

Given that human error is the most important cause of industrial accidents, it seems necessary to identify and analyze human error, assess human reliability, and reduce errors or prevent unfortunate consequences. This study aimed to evaluate human reliability in a petrochemical industry.

**Methods:**

Critical and sensitive jobs were identified by interviewing the staff and supervisors of the industry. Then, the most important human errors and Performance Shaping Factors (PSFs) in each job group were identified. Using the Analytic Hierarchy Process (AHP), PSFs and human errors were weighed and prioritized. Next, the Failure Likelihood Index (FLI) was calculated for each of the human errors identified in the selected tasks. Finally, by converting this index to human error, human reliability was calculated.

**Results:**

Firefighters, site men, and mechanical repairmen had the highest risk and were selected to evaluate human reliability by the AHP-FLI method. Accordingly, six PSFs (training, experience, instruction, stress, task complexity, and environmental conditions) were identified as the most important factors in human error occurrence. The average human error probability was calculated as 0.019, 0.018, and 0.013 in the three job groups of firefighters, site men, and mechanical repairmen, respectively.

**Conclusion:**

This study showed that the AHP-FLI method could be a suitable method for assessing human reliability in the petrochemical industry since it could measure the impact of different PSFs on the probability of human error.

## 1 Introduction

At present, many jobs and processes are considered critical because an error in them can have catastrophic consequences, such as death, severe economic damage, and widespread environmental pollution. One of the critical industries is the oil, gas, and petrochemical industry. According to surveys, over the past 30 years, 400 accidents have resulted in environmental damage and pollution many of which were related to fires and explosions caused by chemical leaks. This also accounted for 80% of all fires and explosions in the chemical industry [1]. One of the most important incidents in this area is the Bhopal disaster, in which more than 500,000 people were in direct contact with methyl isocyanate gas [2]. Similarly, about 100 tons of benzene and nitro-benzene leaked into the Songhua River in China in November 2005, resulting in severe environmental pollution and contamination of drinking water supplies used by more than 10 million people [3]. Studies have shown that human error is responsible for more than 80% of such accidents in the chemical and petrochemical industries [2, 4]. Given the complexity of industrial systems and processes, creation of high-risk technologies and processes, the fact that humans are unpredictable and fallible, and human error is the most important cause of industrial accidents, it seems necessary to identify, predict, and analyze human error, assess human reliability, and devise appropriate control strategies to eliminate and reduce errors or prevent unfortunate consequences. One of the most influential approaches is to examine the interaction between human reliability and human error and the impact of these two categories on each other.

Studies on human reliability analysis have now become one of the essential phases in human and systemic Probability Risk Assessment (PRA) [5]. Human reliability refers to the likelihood that the system activities will be performed by humans correctly and without errors within a specified period of time. The set of methods and models used to predict human error in activities is called Human Reliability Analysis (HRA) [6, 7]. Reliability is a structure influenced by many uncertain factors stemming from various sources, such as design, manufacture, and production [7]. Human error is the most important factor affecting safety because its effect often goes beyond random deviation. Research results have shown that the existing reliability is not in line with the expected reliability, and human error is the main reason for this gap. Human Error Analysis (HEA) is required to calculate the existing reliability.

HEA is often used in the safe operation of nuclear power plants and other complex systems [8, 9]. HRA is performed as a part of a system safety analysis to analyze and predict the human error probability in these industries [10]. One of the most important steps in the human reliability assessment is to identify the factors that affect human performance and can increase the human error probability [5]. In general, human behavior is influenced by PSFs [11]. These factors are divided into three categories, namely external (such as workplace condition, equipment design, and instructions), internal (such as personal skills, experience, excitability, and level of training), and stressors (physiological and psychological stress at work). If the levels of these PSFs are inadequate, they increase the likelihood of human error [12, 13]. A number of HRA techniques have been proposed and are being widely used. These methods include Success Likelihood Index (SLIM), Failure Likelihood Index (FLIM), Paired Comparison (PC), etc. These methods are commonly used to simplify HRA.

Due to the multiplicity of these factors, the multi-criteria decision making (MCDM) can be used to assess reliability. Standard MCDM methods include AHP, analytic network process (ANP), data envelopment analysis (DEA),multi-objective programming, and goal programming.

In this research, a framework that combines various data and implicit preference as in AHP is developed to utilize preference and objective data to tackle the drawbacks of using a particular method alone.

## 2 Literature review

Quantifying Human Error Probability (HEP) is a difficult part of HRA. Although research has been done to quantify HEP, only a few of these techniques have been successfully implemented. Techniques that have been proposed and widely used as tools for HEP estimation include Human Error Assessment and Reduction Technique (HEART), Technique for Human Error-Rate Prediction (THERP), and SLIM. The SLIM has taken many forms since its early development. For example, FLIM is a form of SLIM used in some studies. The FLIM uses the FLI versus the Success Likelihood Index (SLI) [14]. This method has been designed to determine the human error probability, but it is also used to evaluate the PRA. The advantages of this method are its easy application and high flexibility. This method is one of the most important tools used in expert judgment in estimating the HEP [15]. In this method, assessment of the success likelihood of tasks depends on the combined effect of PSFs. The most important advantage of this method, compared to other methods used to assess human reliability, is the selection of PSFs according to the prevailing occupational conditions. In other words, since the working conditions in various jobs are different, PSFs can be selected according to the conditions in that job [16].

In the FLIM, the evaluator can determine the probability of human error for each task by determining the values for the PSFs. In most studies, due to the lack of information resources in the area of HEP, the use of expert judgment methods is highly accepted [17]. However, since these methods are based on expert judgment, they have limitations. The FLIM also uses expert judgment to provide a numerical framework for activities as the input to the probability formula related to human error. On the other hand, given the high dependence of these methods on expert judgments, the results can be influenced by the judgment of any expert, creating limitations such as incompatibility of judgments and difficulty of quantifying the PSFs.

One of the methods used to eliminate the limitations of expert judgment in the FLIM is using MCDM. MCDM methods have evolved to accommodate different types of applications in the literature [18, 19, 20]. Researchers suggest that the trend to use the MCDM method is to combine two or more methods to compensate for the shortcomings in each particular method [21, 22]. Among MCDM, AHP is selected due to its ability in decomposing a decision problem into its fundamental parts, which can be hierarchically structured [23, 24]. Vaidya and Kumar (2006) examined the applications in different fields using the AHP technique. The authors note that future applications of AHP include being widely used for decision making and addressing more complex issues based on an integrated application of AHP and other techniques [18, 21].

One of the important advantages of the AHP method is that it enables group decision making so that it combines the decisions of all group members in such a way that the optimal decision includes the opinion of all members [14]. A detailed description of this method has been provided by Saaty [25]. AHP is based on user experience and judgment and the results are objective [26] and realistic [27, 28].

To make the results of the analysis more reasonable, fuzzy set theory is used. Fuzzy Analytic Hierarchy Process (FAHP) is a combination of fuzzy theory and AHP [29]. The AHP method can be effective in solving the problem when researchers are sure that the opinions given by experts are carefully, harmonious, and proficiently. However, the AHP method used an almost crisp decision-making program which does not take into account the uncertainty of one's judgment. Due to its nature, linguistic values are inconsistent which requires ambiguity to reduce the risk of making wrong decisions [30]. The main focus is that classical method should be used when the information is certain; if the information is not certain, fuzzy method should be preferred [31]. Based on the information obtained from previous studies and the results of in-industry monitoring, and therefore, if the data are certain, AHP is preferred.

There have been a number of studies on the quantification of subjective judgment or the elicitation of subjective probabilities using AHP [32, 33, 34, 35]. These studies have suggested the possibility that AHP can be used to estimate HEPs. Although applications in MCDM have been increasingly used, the evaluation of human reliability considering a framework incorporating different MCDM approaches is scarce. Existing literature were highlighted in Table 1 and the proposed study was discussed as follows:

1. While MCDM methods are found in a wide range of applications in the literature, studies focusing on human reliability assessment are still rare.
2. For the AHP, Satty [43] assumed that the elements in each group of a hierarchy should be independent. For the FLIM, the probability of human error occurring in a particular condition depends on the effects of the PSFs. Therefore, a combination of these two methods can improve the results. AHP-FLIM requires human errors as well as PSFs to be independent.
3. Only one study has been performed using the AHP-FLIM method, which is also in the construction industry and has not been done in more complex industries such as the petrochemical industry.
4. For the first time in Iran, in this study, the factors affecting human error in sensitive and vulnerable jobs in the petrochemical industry were investigated and human errors were determined, prioritized and weighted specifically and in accordance with the working conditions.

**Table 1:** Summary of literature review in human reliability in the industries.

Study	Year	Method	Industry type	Outcome
Blackman et al. [36]	2008	Standardized Plant Analysis Risk Human Reliability Analysis (SPAR-H)	Nuclear Power plant	Quantification Analysis of human reliability and estimation of human error related to operators
Zhou and Kou [14]	2010	AHP-FLIM	Construction	The proposed AHP-FLIM method makes a meticulous analysis of occurrence of HEs in construction.
Sun et al. [37]	2011	Human Cognitive Reliability (HCR)	Airport control tower	The possibility of human error in the scenario for the collision of two aircraft in terms of training level and stress was investigated.
Musharraf et al. [38]	2013	SLIM	Oil rigs	In the emergency response process, the minimum human reliability was when gathering in a safe place.
Zhou et al. [39]	2018	fuzzy logic theory, Bayesian network (BN), and cognitive reliability and error analysis method (CREAM)	Tanker shipping industry	The evaluation of HEP according to the proposed HRA model is very promising and the HRA model is consistent with the original CREAM approach.
Petruni et al. [40]	2019	AHP	Automotive industry	The Analytic Hierarchy Process (AHP) provides a way of assisting safety managers and risk assessors in the HRA technique selection process.
Tavakoli and Nafar [41]	2020	Human Factors Analysis and Classification System (HFACS)	Maintenance team of power transmission system protection	Human error factors are ranked to help improve human reliability.
Ahn and Kurt [42]	2020	CREAM and fuzzy theory	Firefighting procedure	The proposed method can evaluate the context in a maritime scenario based on the CREAM basic method and illustrate practical application to onboard procedures in the context in vessels by using the CREAM extended method.

Considering the points mentioned above, this study aims to evaluate the factors affecting human error in the sensitive and vulnerable jobs of a petrochemical industry and to assess the human reliability of these jobs.

## 3 Materials and methods

In this section, first how to perform the calculations of methods including AHP and FLIM and theoretically and then, how to use these two methods in the form of AHP-FLIM method is stated.

### 3.1 Theory

#### 3.1.1 AHP

The AHP is a multi-criteria decision-making method for complex problems, in which both qualitative and quantitative aspects are considered [26]. What follows is a summary of the steps for performing AHP [44]:

(1) Create a decision hierarchy, break down the problem into a hierarchy of decision elements (Figure 1).

**Figure 1:** Form of decision elements in AHP.
(2) Create judgment data by a pairwise comparison matrix of decision elements. The numerical scale used to assign values to these comparative ratings has been shown in Table 2.

**Table 2:** Value scale for alternative decision comparison.

Scale of relative importance	Definition	Explanation
1	Equally important	Two decisions equally influence the upper-level objective.
3	Moderately important	One decision is moderately more favorable for the upper-level objective fulfillment.
5	Strongly more important	One decision is strongly more favorable for the upper-level objective fulfillment.
7	Very strongly more important	One decision is significantly more favorable for the upper level objective fulfillment.
9	Extremely more important	The difference between the influences of the two decisions is extremely significant.
2, 4, 6, 8	Intermediate judgments value	When a compromise is necessary to give an intermediary judgment among the previous values.
(3) Calculate the priority vector and check the consistency of the matrix.
(4) Calculate the relative weight of the decision elements.
(5) Verify the consistency of the entire hierarchy.

Consistency index (C.I) defines as follow (Eq. (1)):

(1) C.I = λ_max_ – *n* /*n* – 1

where λ_max_ is the maximum eigenvalue of the matrix and *n* is the length of the matrix and C.I is the consistency index. Dividing the value of C.I. by R.I calculates the consistency ratio. If the consistency ratio is less than ten percent, the calculations are approved, otherwise the analysis must be repeated. R.I is a random matrix consistency index, which is calculated from the calculation of consistency index values for matrices whose numbers are completely random.

#### 3.1.2 FLIM

The basic hypothesis of the FLIM is that the HEP is associated with PSFs. PSFs are the parameters that affect the human's ability to complete a given task. Therefore, the first step of the FLIM is to determine the PSFs set. The following are the main steps for implementing the FLIM [45].

(1) Identify the set of PSFs.
(2) Weigh each PSF, *wi* ($\sum_{i=1}^{n}wi$ = 1 = 1; *i* = 1, 2, · · ·, N; N is the number of PSFs), through judgments by experts. Assume the largest value for the most important PSF. PSF weight is the relative importance of a given PSF in comparison to the PSF judged to be the most important. Moreover, the PSFs are ranked in the order of importance.
(3) Rate each task, *ri* (0 ≤ *ri* ≤ 1). Task rating is a measure of the quality relevant to each PSF independent of other PSFs.
(4) Calculate FLI by

(2) $${\text{I}}_{\text{FLI}}=\sum_{i=1}^{n}wi\;ri,\;0\leq {\text{I}}_{FLI}\leq 1$$

where *wi* was the weight calculated for human error in each PSF, *ri* was the PSF weight, and I_FLI_ was the FLI for each error.

(5) Compute HEPs by the following calibration equation

(3) Log PHEP = *a*I_FLI_ + *b*

where *a* and *b* were constant values calculated using the minimum and maximum values of FLI (calculated in the previous step) and their corresponding Basic Human Error Probability (BHEP).

(7) Identify uncertainty bounds and check judgment consistency.

The execution of this method has been described in details in the study conducted by Zimolong et al. [45]. The assessor can utilize the expert judgment technique when the reference tasks are unavailable. In Eq. (2), FLI and the objective probability agree with the exponential relationship [46].

### 3.2 Study process

For problems arising from the judgment of experts in FLIM, including inconsistencies in judgment and the difficulty in roundly considering relevant PSFs, the consistency of all measurements and judgments can be examined in AHP [14] and FLIM can consider PSFs successfully. The HE systematic reliability analysis method should focus on the FLIM along with AHP. The FLIM was used to extract the FLI of the target task. The AHP is used to convert FLI to HEP. By applying this method in HEA, the above problem can be overcome and HEPs can be calculated easily and quickly.

This cross-sectional descriptive study aimed to evaluate the human reliability of critical and sensitive jobs of a petrochemical industry located in South Pars Special Area, Iran using AHP-FLIM. The stages of the study have been shown in Figure 2.

**Figure 2:** The study process.

#### 3.2.1 Identifying critical jobs sensitive to human error

At this stage, after visiting the desired industry and interviewing and consulting with the staff and supervisors, all job groups within the petrochemical company were identified. Then, using risk number (accident severity × accident frequency), critical and sensitive jobs were selected. Based on the number of risk, it is possible to identify jobs in which accidents are more likely to occur (i.e. sensitive and critical jobs).

#### 3.2.2 Identifying human errors in critical and sensitive jobs

The most likely human errors in each job were identified by interviewing six personnel and six supervisors in each critical and sensitive job.

#### 3.2.3 Identification PSFs

Six personnel and six supervisors for each critical job selected in the previous phase were asked to identify the most important factors affecting human error in their jobs among ‘skill’, ‘experience’, ‘training’, ‘environmental conditions’, ‘task complexity’, ‘stress’, ‘equipment design’, ‘time pressure’, and ‘instructions’. It should be mentioned that these nine PSFs are among the most important factors affecting human error, which have been mentioned in several studies.

#### 3.2.4 Prioritization of PSFs using AHP

The goal of this section was prioritization and weighting of PSFs. So, there were 6 criteria. To do this, the PSFs were compared in pairs using an expert questionnaire. To weigh the pairs of comparisons, 12 individuals including six safety experts and six operators were asked to prioritize the PSFs using a comparative weighting table (Table 2). The given weights were then transferred to the paired comparison matrix of the PSFs. At the end of this step, the relative importance and weight of each PSF in the occurrence of human error in each job were determined using the Super Decision software. It should be noted that the consistency ratio was less than 10%.

It is important to select the right experts in this method. They were required to have professional experience and knowledge in this field. The safety experts' group consisted of 3 Ph.D. candidates, and 3 professors. They have majored in occupational safety and were familiar with AHP and FLIM. The average work experience of selected operators in petrochemical management was 5 years.

#### 3.2.5 Prioritization of human errors in each PSF using AHP

In order to prioritize human errors in selected jobs (critical jobs selected in the previous steps), AHP method was used. At this stage, the relative probability of human errors identified for each PSF was determined using AHP. In so doing, the identified human errors were compared in pairs using an expert questionnaire. Afterwards, the weight of human errors in each PSF was determined using the relative weighting table and was transferred to the human error paired comparison matrix. Then, the relative importance and weight of each error in each PSF were determined using the AHP method and the Super Decision software. It should be noted that the consistency ratio was less than 10% (Figure 3).

**Figure 3:** The evaluation framework for prioritization of human error.

#### 3.2.6 Calculating the HEP and human reliability for each of the human errors using FLIM

The FLI for each of the errors identified was calculated using Eq. (2). The I_FLI_ of each error was estimated separately for all members including the two groups (six safety experts and six operators). Then, the geometric mean was reported as the final FLI for each error. The FLI was converted to HEP using Eq. (3) [43]. After determining the HEP, the average probability of human error was calculated and human reliability in each job group was determined using Eq. (4).

(4) R = 1 – P

Where R was human reliability and P was the average probability of human error in each occupational group.

## 4 Results

The results of the various stages of the study have been described below.

### 4.1 Identifying critical jobs sensitive to human error

The results of choosing jobs in the industry in terms of the degree of susceptibility and vulnerability to human error have been presented in Table 3. Accordingly, from the eight jobs in the industry (board men, site men, firefighters, office workers, mechanical repairmen, service workers, HSE men, and storekeepers), firefighters (n = 27), site men (n = 90), and mechanical repairmen (n = 26) had the highest accident risk and were selected to evaluate human reliability by the AHP-FLIM. The mean age (standard deviation) of the selected job groups was 33 [8], 30 [6], and 27 [4] years, respectively. Besides, their mean work experience (standard deviation) was 8 [5], 6 [5], and 6 [4] years, respectively.

**Table 3:** Prioritization of jobs in the petrochemical industry studied by the rate of accident risk due to human error.

Factors	Jobs						
	Storekeepers	HSE men	Service workers	Mechanical repairmen	Office workers	Firefighters	Site men
Severity of the accident	0.107	0.087	0.054	0.302	0.046	0.128	0.273
Probability of the accident	0.083	0.07	0.067	0.283	0.051	0.163	0.28
Risk rate (severity × probability)	0.008	0.006	0.003	0.085	0.002	0.020	0.076

### 4.2 Identifying human errors in critical and sensitive jobs

The most important human errors along with their descriptions and consequences have been listed in Table 4. Accordingly, “negligence in wearing personal protective equipment” was a common mistake in all the three occupational groups. Indeed, “gas testing in the wrong place” was reported among firefighters and site men.

**Table 4:** Human errors identified in the critical job groups in the petrochemical industry.

Error code	Task	Error description	Consequences
Firefighters			
Ef.1	Wearing personal protective equipment (PPEs)	Forgetting to wear PPEs	Probability of injury and even death during operations
Ef.2	Fire extinguishing	Fire extinguishing operations are carried out with inadequate or wrong equipment	Delay in firefighting resulting in escalation of life and financial losses
Ef.3	Gas testing using the device	The operator does gas testing in the wrong place	The gas testing has not been operated properly, resulting in the possibility of explosion and fire at work
Ef.4	Fix leakage	No fix leakage operations done	Probability of fire and explosion due to sparks or poisoning with toxic gases
Ef.5	Permit to work review to know the safety principles during operation	Incorrect interpretation of the information contained in the permit to work	Possibility of personal injury due to lack of knowledge about safety principles
Ef.6	Dispatch to the accident place	The firefighters arrive late	Fire extinguishing delay and escalation of damage
Ef.7	Disconnection of input energy from equipment	Disconnection of input energy from equipment is not performed prior to Extinguishing operations.	The occurrence of accident resulting in a delay in extinguishing and intensifying damage
Site men			
Es.1	Wearing personal protective equipment (PPEs)	Forgetting to wear PPEs	Probability of injury and even death during operations
Es.2	Checking for non-greasy protective clothing before working on the oxygen line	Checking for non-greasy protective clothing before working on the oxygen line is not done.	Because of the clothes being greasy and exposed to oxygen, there is a possibility of explosion during work.
Es.3	Use of cast iron equipment when working on gas lines	The use of cast iron equipment is forgotten.	There is a possibility of explosion due to spark during work.
Es.4	Permit to work review to know safety principles when entering reactors and converters	Incorrect interpretation of the information contained in the permit to work	Possibility of personal injury due to lack of knowledge about safety principles
Es.5	Gas testing using the device	The operator does gas testing in the wrong place	The gas testing has not been operated properly, resulting in the possibility of explosion and fire at work
Es.6	Torching	Torch operation is performed in an incorrect sequence	The unit may be destroyed and there may be heavy financial losses.
Es.7	Hot spot test∗	Hot spot test is not done.	The temperature is increased in high-pressure converters, which results in the possibility of fire and explosion.
Mechanical repairmen			
Em.1	Wearing personal protective equipment (PPEs)	Forgetting to wear PPEs	Probability of injury and even death during operations
Em.2	Checking that the bolts are not greasy before placing them on the oxygen line	Bolts are not checked before being placed on the oxygen line.	The explosion is likely to occur due to the greasiness of the bolts and their contact with oxygen.
Em.3	Checking for non-greasy protective clothing before working on the oxygen line.	Checking for non-greasy protective clothing before working on the oxygen line is not done.	Because of the clothes being greasy and exposed to oxygen, there is a possibility of explosion during work.
Em.4	Fixing leaks from the serving line	Fixing leaks from the line is not done	Probability of fire and explosion due to sparks or poisoning with toxic gases
Em.5	Using non-bronze tools during leakage removal	The use of non-bronze tools is forgotten.	Probability of fire and explosion due to sparks.
Em.6	Installing the control valve	The control valve is installed in the wrong direction.	Improper installation of the control valve increases the pressure in the system and may cause the connection pipe to break.
Em.7	Closing the flange washer.	Closing the flange washer is forgotten.	Failure to close the washer can lead to material leakage and can cause an explosion.

∗ Hot spot test is performed to check the resistance status of high pressure converters. In these converters, excessive temperature rise can lead to the loss of the converters resistance and eventually melting.

### 4.3 Identification and prioritization of PSFs

Out of 9 PSFs, workers chose 6 PSFs as the most important factors including stress, task complexity, experience, training, instruction, and environmental condition. Then these PSFs entered the AHP as criteria.

PSFs and their prioritization results in critical and sensitive occupational groups in terms of the weights have been presented in Table 5. Accordingly, the lowest AHP weights in the PSFs of firefighters, site men, and mechanical repairmen were related to task complexity (0.051), task complexity (0.065), and stress (0.057). On the other hand, the highest AHP weight in firefighters, site men, and mechanical repairmen was related to training (0.420, 0.408, and 0.412, respectively).

**Table 5:** Prioritization of PSFs by the AHP method in critical and sensitive job groups in the petrochemical industry.

PSFs	Job group					
	Mechanical repairmen		Site men		Firefighters	
	Non-normalized weight	Normalized weight	Non-normalized weight	Normalized weight	Non-normalized weight	Normalized weight
Stress	0.028	0.057	0.034	0.069	0.039	0.079
Task complexity	0.041	0.083	0.032	0.065	0.025	0.051
Experience	0.118	0.236	0.152	0.304	0.153	0.306
Training	0.206	0.412	0.204	0.408	0.210	0.420
Instruction	0.068	0.136	0.039	0.079	0.037	0.074
Environmental conditions	0.036	0.072	0.036	0.072	0.033	0.067

### 4.4 Prioritization of human errors

The prioritization of errors by the AHP method in critical and sensitive job groups has been illustrated in Table 6. In fact, for each job, 7 human errors were include in the AHP as criteria. As seen, the highest and lowest mean weights determined for the firefighters were related to Ef.3 error (0.228) and Ef.6 error (0.054), respectively. The highest and lowest mean weights determined for the site men were related to Es.3 error (0.0300) and Es.7 error (0.061), respectively. Finally, the highest and lowest mean weights for mechanical repairmen were related to Em.4 error (0.361) and Em.5 error (0.060), respectively.

**Table 6:** Prioritization of human errors by the AHP method in critical and sensitive job groups in the petrochemical industry.

Mechanical repairmen			Site men			Firefighters		
Error code	Non-normalized weight	Normalized weight	Error code	Non-normalized weight	Normalized weight	Error code	Non-normalized weight	Normalized weight
Em.1	0.041	0.082	Es.1	0.030	0.061	Ef.1	0.031	0.062
Em.2	0.045	0.090	Es.2	0.056	0.112	Ef.2	0.042	0.084
Em.3	0.059	0.118	Es.3	0.033	0.066	Ef.3	0.142	0.284
Em.4	0.180	0.361	Es.4	0.148	0.296	Ef.4	0.117	0.234
Em.5	0.030	0.060	Es.5	0.150	0.300	Ef.5	0.110	0.221
Em.6	0.087	0.175	Es.6	0.035	0.070	Ef.6	0.110	0.221
Em.7	0.055	0.110	Es.7	0.045	0.091	Ef.7	0.027	0.058

### 4.5 Calculating the FLI and assessment of human reliability in the study groups

The FLI for each of the identified human errors, results of the calculation of HEP, and human reliability for each identified human error in the job groups have been presented in Table 7. Accordingly, the highest FLI was related to the error Ef.3 (The operator does gas testing in the wrong place) for the firefighters, error Es.5 (The operator does gas testing in the wrong place) for the site men, and error Em.4 (Fixing leaks from the line is not done) for the repairmen. The average HEPs for firefighters, site men, and mechanical repairmen were 0.019, 0.018, and 0.013, respectively.

**Table 7:** The FLI for human errors, HEP, and human reliability assessment (R) in critical and sensitive job groups in the petrochemical industry.

Mechanical repairmen				Site men				Firefighters			
Error code	FLI	HEP	R	Error code	FLI	HEP	R	Error code	FLI	HEP	R
Em.1	0.078	0.010	0.989	Es.1	0.057	0.009	0.009	Ef.1	0.059	0.010	0.989
Em.2	0.088	0.011	0.988	Es.2	0.109	0.013	0.986	Ef.2	0.081	0.011	0.988
Em.3	0.114	0.012	0.987	Es.3	0.063	0.010	0.989	Ef.3	0.281	0.039	0.960
Em.4	0.356	0.029	0.970	Es.4	0.292	0.038	0.961	Ef.4	0.23	0.028	0.971
Em.5	0.057	0.009	0.990	Es.5	0.296	0.039	0.960	Ef.5	0.217	0.026	0.973
Em.6	0.168	0.014	0.985	Es.6	0.067	0.010	0.989	Ef.6	0.054	0.0098	0.9901
Em.7	0.106	0.011	0.988	Es.7	0.088	0.011	0.988	Ef.7	0.050	0.0095	0.9904
Mean of human error probability			0.013	Mean of human error probability			0.018	Mean of human error probability			0.019
Mean of human reliability			0.987	Mean of human reliability			0.982	Mean of human reliability			0.981

## 5 Discussion

In the present study, the AHP-FLIM was used to determine human reliability in critical and sensitive jobs of a petrochemical industry in Iran. Sensitive and critical jobs were identified by conducting AHP for all job groups in the petrochemical industry. Accordingly, three occupational groups, namely repairmen (risk = 0.085), site men (risk = 0.076), and firefighters (risk = 0.02), were found to be critical and sensitive jobs in terms of human error occurrence.

There were common human errors in the critical and sensitive jobs of this study. Finding ways to reduce these errors can be a good way to reduce the risks of major accidents in the petrochemical industry. One of these errors was “not using personal protective equipment”. Although the probability of this error was low in all three job groups, due to the widespread perpetration of this error by the personnel and the importance of using personal protective equipment, attention needs to be paid. Not using personal protective equipment has always been a major cause of injury to workers. For example, according to the Iranian accident statistics, ‘the use of hazardous clothing’ that is only one part of ‘not using personal protective equipment’ has always been a major cause of occupational accidents [47]. During the first six months of 2010, 778 people died from work accidents, indicating an 18.8% increase compared to the same period in 2009. Lack of safety considerations as well as negligence in the use of safety equipment and personal protective equipment played a major role in the occurrence of these accidents [48].

Another important issue in the area of common errors was gas testing. According to the US Chemical Safety and Hazard Investigation Board (CSB) investigations since 1990, more than 60 deaths from fires and explosions caused by work in hot environments occurred in 11 accidents. The main causes of these accidents were “failure to perform gas testing” (A.V. Thomas accident in 2009, Mar Oil accident in 2008, and Philipi Services accident in 2008) or “inappropriate gas testing” (TEPPCO accident in 2009, Penzzoil Refinery accident in 1995, and Motiva Enterprises accident in 2001), indicating the important role of human error in gas testing in the occurrence of accidents [49]. According to Table 7, the error “Operator does gas testing in the wrong place” with the probability of 0.039 was identified as the most important error among the firefighters and site men. Evidence has indicated that new staff at the petrochemical industry are offered a short training course on the principles of performing gas testing correctly and the risks involved in this task. This course is only for beginners, and retraining courses are not held during their employment in order to raise their awareness about the very high sensitivity of this task and its risks as well as to update their information. Therefore, due to the importance of gas testing, periodic and scheduled retraining sessions are recommended to be held during the work experience. Moreover, the gas testing instructions in the firefighting department are very general and somewhat vague. For example, by changing the gas meter model, the changes in the instructions are either delayed or not done. Hence, appropriate instructions should be provided in clear details. In order to recover and remediate this human error, it is recommended to repeat the gas test by more than one person in the environment.

Permit to work system in the sensitive jobs of the petrochemical industry was also susceptible to human error. Permit to work system is one of the most important safety systems in preventing accidents during repairing work and is one of the most sensitive and susceptible occupational tasks to human error. For example, one of the main causes of the Piper Alpha accident was the failure in permit to work during shift delivery. The failure in permit to work was also the main cause of the Hickson accident in 1992 [50]. In the current study, “Incorrect interpretation of the information contained in the permit to work” with the probability of 0.038 and a slight difference from “Operator does gas testing in the wrong place” was identified as the second major error among the site men (Table 7). According to the study carried out by Jahangiri et al., the following suggestions were made to reduce the likelihood of this error: 1. Employing a qualified person for gas testing (except for site men); this can reduce the dependency level of the tasks conducted by site men, 2. Providing a specific appropriate procedure for the task of “flammable gas testing”, 3. Revising the permit to work procedure for detailed explanation of the responsibilities of all the operators involved in permit to work issuance and its related work activities, and 4. The automation of the permit to work issuance procedure as a simple and appropriate solution can be very effective in preventing and reducing the probability of human errors [50].

Based on Table 7, the “Fixing leaks from the line is not done” error with the probability of 0.029 was found to be the most important human error in the mechanical repair job group. In the petrochemical industry studied, the personnel employed in the mechanical repair unit are a part of the contractual force and do not receive specialized training after being recruited. As most of the staff in this unit have low levels of education, they require specialized training in order to perform critical tasks such as fixing leaks from the serving line. The guidelines for this task also refer to continuing education and training, but only one general training course is initially held in the industry. Furthermore, the instructions on how to repair a leak in the repair unit are somewhat vague and need more clarification. On the other hand, due to the lack of knowledge and expertise in the “fixing leak” task, high stress loads on the individuals can affect their performance. Given the inverse relationship between high occupational stress and the ability to do work, high levels of human error are likely in these individuals. It is recommended that the workers be periodically trained on how to fix leaks and service the line. Also, the presence of a supervisor during the inspection and elimination of leaks, in addition to checking the proper performance of the task, can help reduce stress.

Among the PSFs identified in the present study, “training” was identified as the most important factor affecting human error occurrence in all three job groups. Studies have shown that low levels of education increased the likelihood of human error [51]. In these tasks, employees are often in situations where they do not have access to signs and instructions and have to rely on their vigilance and take initiatives to solve problems. Obviously, not having sufficient knowledge increases the probability of human error [52]. In other words, most accidents occur when a person is asked to perform a task while s/he lacks the technical and empirical competence to perform it [52]. In case the workers' technical capabilities do not meet their job requirements, it causes safety and health problems, reduces productivity, and increases accidents and the associated costs [53]. Staff training is essential to change people's attitudes towards development of safe behaviors [54, 55]. In fact, staff training is a key element in the development of safe behaviors, which results in the creation of a safe working environment [56].

Experience was identified as the second most influential factor in the occurrence of human error in all three job groups. The reason for the distinction between education and experience is the source of knowledge. Training is often done through published contents and is generally called the ‘book-based’ debriefing style. However, experience includes other resources, such as skills. This type of knowledge is acquired when the individual is placed in a particular practical situation. Human experience is one of the most effective factors in reducing human error. Experienced people are more familiar with equipment and workplaces and can make the right decisions in specific situations more quickly [57].

## 6 Conclusion

The results of this study showed that the AHP-FLIM could be used to analyze and quantify the potential errors, evaluate human reliability, and devise appropriate control strategies to eliminate and reduce the errors or prevent the unfortunate consequences in critical jobs of petrochemical industries. In addition to assessing the impact of different PSFs on HEP, AHP-FLIM can determine PSFs according to the workplace conditions. Given the above points, this method can be used in the studies concerning human reliability in petrochemical industries. It is suggested that in future research, this method be used to quantify the relationship between human reliability and individual characteristics in the petrochemical industry.

## Declarations

### Author contribution statement

Asma Zare: Conceived and designed the experiments; Analyzed and interpreted the data; Wrote the paper.

Naser Hoboubi: Performed the experiments; Analyzed and interpreted the data; Wrote the paper.

Salman Farahbakhsh: Analyzed and interpreted the data; Wrote the paper.

Mehdi Jahangiri: Conceived and designed the experiments; Contributed reagents, materials, analysis tools or data.

### Funding statement

Mehdi Jahangiri was supported by 10.13039/501100004320Shiraz University of Medical Sciences [937086].

### Data availability statement

Data included in article/supplementary material/referenced in article.

### Declaration of interests statement

The authors declare no conflict of interest.

### Additional information

No additional information is available for this paper.
